The article "Influential Usage of Big Data and Artificial Intelligence in Healthcare" was retracted in 2023. Reasons: signs of a paper mill; suspected computer-generated content; unreliable results or conclusions; concerns about the data.

# Influential Usage of Big Data and Artificial Intelligence in Healthcare

**DOI:** 10.1155/2021/5812499

**Published:** 2021-09-06

**Authors:** Yan Cheng Yang, Saad Ul Islam, Asra Noor, Sadia Khan, Waseem Afsar, Shah Nazir

**Affiliations:** ^1^Foreign Language Department, Luoyang Institute of Science and Technology, Luoyang, Henan, China; ^2^Foreign Language Department/Language and Cognition Center, Hunan University, Changsha, Hunan, China; ^3^Department of Computer Science, University of Swabi, Swabi, Pakistan

## Abstract

Artificial intelligence (AI) is making computer systems capable of executing human brain tasks in many fields in all aspects of daily life. The enhancement in information and communications technology (ICT) has indisputably improved the quality of people's lives around the globe. Especially, ICT has led to a very needy and tremendous improvement in the health sector which is commonly known as electronic health (eHealth) and medical health (mHealth). Deep machine learning and AI approaches are commonly presented in many applications using big data, which consists of all relevant data about the medical health and diseases which a model can access at the time of execution or diagnosis of diseases. For example, cardiovascular imaging has now accurate imaging combined with big data from the eHealth record and pathology to better characterize the disease and personalized therapy. In clinical work and imaging, cancer care is getting improved by knowing the tumor biology and helping in the implementation of precision medicine. The Markov model is used to extract new approaches for leveraging cancer. In this paper, we have reviewed existing research relevant to eHealth and mHealth where various models are discussed which uses big data for the diagnosis and healthcare system. This paper summarizes the recent promising applications of AI and big data in medical health and electronic health, which have potentially added value to diagnosis and patient care.

## 1. Introduction

AI is a field of computer science, which is capable of copying human characteristics, capacity of learning, and storage of knowledge. It executes human brain tasks in most of the fields in all aspects of our daily life using big data applications. Super computers are analyzing big data using the algorithms of advanced deep learning machines, which has allowed the improvement of output in the field. This field has led very needy and tremendous enhancement in every field of life, especially in healthcare. Big data analysis is entered in biomedical sciences; the foremost source of big data has been discussed and explained, especially in oncology, cardiovascular disease, allergic diseases, clinical work, ear diseases, and so on. Along with this, it also touches some aspects of need to combine several pathological and clinical sources and quality of life data [1] as well as the unprecedented and quantitative datasets of neuroscience [2]. Medical care and treatment are getting enhanced day by day. Researchers are collecting data to make human care and diagnosis disease efficiently and operationally. Medical doctors are skeptical about the help that artificial intelligence can deliver to them in their medical practices. Studies have explored an understandable experience which includes all challenges, risks, and comfort since the implementation of AI programmed with the help of big data in healthcare within a contagious disease setting. The aim of the program was at designing a set of tools which can support an accurate, objective, and clinical decision-making process efficiently [3]. In biomedicine, there are many ways to collect data from observation and experiments. Scientists are often struggling to collect data about the disease and on how data are being generated for the treatment of disease. This biomedical information is to create thinking, managing, and analyzing and the way they can transform into further scientific perception for enhancing patient care. This is the major challenge for the National Institutes of Healthcare (NIH) to lead the big data to knowledge representation. The agencies are making efforts to collect increasingly data with increasing research productivity. Leading centers are developing to handle this type of cases with large-scale data. They are going to research how much accurate equipment is required for the new generation of biomedical data scientists. In today's world, NIH and Big Data to Knowledge (BD2K) seek the position of data sciences in biomedical research [4].

The article "Influential Usage of Big Data and Artificial Intelligence in Healthcare" was retracted in 2023. Reasons: signs of a paper mill; suspected computer-generated content; unreliable results or conclusions; concerns about the data.

Health information technology is designed due to the solution of complex problems such as health disparities. Mix results can be obtained by demonstrating a direct impact on health outcomes. For all these, we must know about collective intelligence, big data, informatics capacities, corresponding terms of smart health, knowledge exchange knowledge, ecosystem, and situational awareness. Standards, guidelines, and objections are established by public health informatics for health equity and health disparities, which will increase health literacy and access to care [5]. Fodeh and Zeng [6] have presented the notation of big data which is used for three words: volume, variety, and velocity. This is the foremost concept which is associated with the dimension's volume, and the variety is very relevant to the biomedical data gained by patients, including tabulated and structured data. The biomedical research communities are struggling to escalate in the clustering and analysis of big data. Mining big data probably holds plenty of information and has a possible way and source for giving knowledge; data mining and machine learning methods are useful for such data series in a challenging task. Kavakiotis et al. [7] have discussed a lot of data on advance technologies which are feasible for medical persons. Researchers have led a lot of research on diseases like diabetes mellitus, concerning the different types of datasets that are mainly used. These hypotheses will lead us about the various knowledge of technologies and diseases in the world. One should have sufficient data and knowledge about machines and technology before using it, as most of the machines used in medical and healthcare emit radiation which is quite harmful and dangerous for humans and buildings. The proof of principle has been provided for lung cancers which has been collected from five locations. The euroCAT infrastructure has successfully implemented as a radiation clinic. Radiation oncology is facilitated as a euroCAT network and will facilitate the machine [8]. In daily clinical work, imaging data usage has the ability to improve cancer care by knowing tumor biology and helping in the implementation of precision medicine. For accession of the tumor and its microenvironment, radiomics helps in monitoring and evaluating the tumor features such as temporal and spatial heterogeneity.

Limkin et al. [9] have provided a study case which assists in ensuring the actual development and enhancement of radiomics as a biomarker and facilitating its implementation in clinical practice. Gebremeskel et al. have proposed a data mining technique of optimization for envisioning of knowledge extraction by examining clinical datasets to define the decisive features using modeling techniques, capable of handling and analyzing large-scale data in its context [10]. In the analysis, guidelines for using AI to speed up the drug's recovery, so that AI's vision is not strong but important, were used. The rapid development, power, and problem of AI and network medicine technology have speed up the development of treatment in healthcare. The study is a strong proof for the use of AI-assisted tools for drugs and repayment for human diseases, including COVID-19 in times of fatal disease [11]. Various studies have been considered for the qualitative analysis of the COVID-19 [12–14]. These studies have mainly considered corona virus from different perspectives.

The exposure of corona virus disease 2019 puts an increasing burden on the healthcare system. While infected patients have nonserious signs, which can be handled at home, some people develop serious symptoms and need to be hospitalized. That is why it is important to effectively evaluate the severity of COVID-19 and identify the hospital's priorities. COVID-19 has been published in a number of countries in the short term. By choosing a session as a time of patient discharge, including rescue techniques and statistical analysis, it is time to seriously prepare it for decision makers to be prepared for more hospital burden. A cube model was proposed to validate and verify the actual and confirmed cases and deaths, which was then accepted by the World Health Organization. Often during the cholera disease, this research-assisted pairing can be learned. Four diagnostic models, including lymphocytes, lactate dehydrogenase, C-reactive proteins, and neutrophils, have been developed and validated using the XGBoost algorithm [15–17].

The article "Influential Usage of Big Data and Artificial Intelligence in Healthcare" was retracted in 2023. Reasons: signs of a paper mill; suspected computer-generated content; unreliable results or conclusions; concerns about the data.

The contribution of the proposed research is to review the existing research associated to eHealth and mHealth where various models are discussed. The approaches along with the uses of big data for diagnosis of disease in healthcare system are elaborated. The study summarizes the recent promising applications of AI and big data in medical health and electronic health. The study will possibly add value to the research in diagnosis and patient care.

This paper is structured as follows: Section 2 shows the related work to the planned research. Details regarding the applications of big data and AI are given briefly in Section 3. Challenges and barriers faced by healthcare are shown in Section 4. The conclusion of the paper is given in Section 5.

## 2. Literature Review

Miller et al. [18] have presented an overview of biomedical data for the derivation of new knowledge on how clinical decision support tools can be developed from the wealth of available data to modernize clinical care and scientific research of diseases related to neurodegeneration in the precision medicine era. Garcia-Ceja et al. [19] have surveyed sensor data and machine learning about mental health monitoring systems. The main focus of the study is about mental disorders or conditions like stress, anxiety, depression, and bipolar disorder. It is suggested to guide the review of the related categorization taxonomy study and present the overall phase of MHMS. Digital health technologies allow access to optimize clinical care delivery and clinical research to access the information about age of healthcare. Despite the usage of such technologies in research and clinical care faces issues such as data quality, privacy, and regulatory, etc. Sharma et al. [20] summarizes think tank meeting proceedings with goals to delineate a framework for appropriately using digital health technologies in research and healthcare delivery. In Alzheimer's disease (AD), clinical development programs have failed to modify new diseases and to establish quality work instrument for the treatment of new and advanced diseases. The report is based on computer modeling and simulation, which plays a role of being powerful and observational in AD research [21]. Super computers are analyzing big data using algorithms of advanced deep learning machines which have allowed the improvement of output like visual image interpretation to formerly imperceptible levels and promised to change the practice of medicine. AI is a well-known field about what everyone is aware of; it is bringing a tremendous progress in such fields like automation of clinical decisions, disease detectors, imaging analysis in medical diagnosis classifiers, an interventional procedures, and it has the strength to significantly affect the practice interventional cardiology. This distinctive nature of interventional cardiology has made it a supreme target for the evolution of artificial intelligence-based approaches which are delineated to enhance real-time clinical decision making, the elegant flow of work in laboratories, and standardized catheter-based procedures using advance robotics. This study highlights the scope of artificial intelligence, its potential applications, and limitations in interventional cardiology [22].

The article "Influential Usage of Big Data and Artificial Intelligence in Healthcare" was retracted in 2023. Reasons: signs of a paper mill; suspected computer-generated content; unreliable results or conclusions; concerns about the data.

The healthcare domain has obtained its effect by the influence of big data since the sources elaborated in the institutions of healthcare are familiar for their dimensions, heterogenous complication, and excessive spirit. Big data's analytical techniques, tools, and platforms are perceived among numerous fields; their effect on healthcare institutions for fulfilling novel use cases for possible healthcare applications shows promising research directions. In this circumstance, the success of these applications is completely dependent on the fundamental architecture and optimization of suitable and proper tools as signified by introducing research attempts. Palanisamy and Thirunavukarasu [23] have discussed many analytical areas that endure in the patient care system from stockholders' perspectives and appraise big data structure with respect to fundamental data sources, systematic capabilities, and application fields, while the intimation of big data that aids in the development of healthcare ecosystem is also discussed. The modern technique, hidden Markov model (HMM), can be used to manage massive data; the inference of the reproducible and interpretable dynamic brain network can be made possible in different dataset ranges including various other tasks [24]. The previous enhancements in ICT have indisputably improved the quality of people's lives around the globe. Computer technology has led to very needy and tremendous enhancement in the health sector which is commonly known as eHealth (electronic health). For optimizing the full and admirable benefits of this development, it is important to implement it in a cloud-based environment. Beside numerous and elegant benefits of eHealth in cloud computing, its full optimization is still obstructed by facing some challenges like privacy and security. The study mainly focuses on contemporary literatures of many techniques, and the mechanism is used to control privacy and security-related matters in eHealth. The robustness and fragility of these approaches were vocalized. 110 articles were reviewed, and several models were figured out in which solutions were adopted in it. These models were compared, and the articles were reviewed in which a standard and acceptable definition of eHealth was given as it was recommended. Privacy and security requirements were also discussed and provided as per the recommendation of the Health Insurance Portability and Accountability Act (HIPAA). Finally, a dependable and secured architecture for eHealth was proposed that could guarantee the effective, regulated, and dependable access framework to health information [25]. It has also applications in speech and language therapy. However, these therapies are often less willingly available for a few months after stroke. Palmer et al. [26] have assessed a self-managed computerized speech and language therapy (CSLT) aiming to deliver more therapy to patients than they can access through usual care alone. CSLT plus usual care significantly improved in individually relevant word findings, but they did not improve in conversation. Schoettler et al. [27] have presented a review of genome-wide association studies (GWASs) of asthma and those related to allergies, in which he concluded that childhood asthma is correlated to the most independent locus compared with other specified groups of allergic and asthma cases, while adult asthma is correlated to fewer genes which can be considered as a subset of those similar with childhood asthma.

The article "Influential Usage of Big Data and Artificial Intelligence in Healthcare" was retracted in 2023. Reasons: signs of a paper mill; suspected computer-generated content; unreliable results or conclusions; concerns about the data.

## 3. Applications of Big Data and AI

A lot of data in the world is available in different hospitals and healthcare centers, which are collected from disease-affected humans. The amount of this data is increasing day by day [28]. Researchers are trying to analyze the data and extract the diseases that affect the human body. Pobiruchin et al. [29] have extracted new approaches for leveraging cancer in the development of Markov Models, from which the researchers easily extract the clinical patient of breast cancer, which can be easily used for freshly affected bodies in the real world. The study has mainly focused on publishing research on breast cancer, which is concerned with the clinical study of data. In this registry, normally, the patient is covered for 8 years from the clinical registry report. Using the Markov model is very good for creating a good opportunity to make a future planning in the existence of data in healthcare and clinical centers. This is useful to get an easy way to identify the patients and their affections in the future. A deep rule-based fuzzy system is used for accurate mortality rate prediction in hospital intensive care units (ICU'S). In pursuant to this approach, in each base building unit of DRBFS, the same system of input has to be kept. In first 48 hours in ICU, with heterogeneous featuring a set of admissions were extracted for mortality rate in hospital [30]. With data concerned to the health records, recurrent neural networks were used for disease risk prediction. The model results were better for small datasets, whereas for large-scale ones, the concerned model and its application to different patients across the population throughout hospitals were not evaluated [31]. Epidemiologist is using electronic health records which assist evidence provision for interval guidelines and screening intervals while censoring interval and undiagnosed sickness make a path to issues like substantial analytic risk estimation which cannot be addressed by using Kaplan-Meier methods [32]. Zhao et al. [33] have determined the illustration of temporal data in electronic health record (EHR); there were several methods based on symbolic sequence representation of time series data, which can be used in several ways, while several evidence relies on the standard of symbolic sequence representation by comparing it to particular orders initiated by clinical experts with the use of domain knowledge. In various other applications of big data based on trajectory data, the regular behavior of private cars is extracted [34–36].

### 3.1. Disease Prediction and Big Data

Big data and artificial intelligence approaches are commonly presented in mHealth and eHealth applications for self-management and home care of many long-term health conditions. Adaptation of these applications for self-management in asthma multifactorial persistent diseases needs validation and evaluation in real-life setups along with the enhancement of the patient level to personalize predictions concerning the control status of asthma and increasing pitfalls. The study presents a short-term prophecy technique for controlling the asthma status, where multiple categorization models are considered trains for each observed framework along with obligatory preprocessing techniques to improve strength and effectiveness. The support vector machine, random forests, Bayesian network, and AdaBoost are considered machine learning algorithms used in this review [37]. Xin-Di et al. [38] have composed 252 formulae from the synopsis of prescriptions of the Golden Chamber and a treatise on exogenous febrile disease, looking to identify the basic rules dominating the choosing of herbal mixtures by probability models and big data technology. Pashazadeh and Navimipour [39] have provided a detailed and systematic review of the modern mechanisms related to healthcare applications in big data fields. Five of the discussed categories are heuristic based, hybrid mechanism, machine learning, cloud based, and agent based. Harous et al. [40] have enlightened the applications of big data for obesity management using sensory and social data in mobile health architecture, which are mainly proposed for assessing, detecting, and controlling obesity, which depend on a mobile phone to be used for complex operations and processing of the data collected. Using this newly developed mobile architecture, one can tackle the challenges of obesity control, monitoring, and prevention. Different algorithms have been used to generate featured suggestions, recommendations, and warnings to control obesity and its related diseases. In the context of large datasets of physical growth measurements which are regularly used by health professionals, this paper is aimed at regenerating a new growth chart for French children. 32 random primary care pediatricians and 10 volunteer general practitioners were selected across the French main regions where the electronic medical record software was used. All data of physical growth was extracted for pediatric patients with anonymization. A new growth chart was derived which was then compared with the WHO chart and found it correct and error free [41].

The article "Influential Usage of Big Data and Artificial Intelligence in Healthcare" was retracted in 2023. Reasons: signs of a paper mill; suspected computer-generated content; unreliable results or conclusions; concerns about the data.

Mechanical therapies are primarily prescribed for motor, duodenal, endocrine, urinary, respiratory, digestive, neural, and cardiovascular diseases. The speedy evolution of healthcare is driven by the enhancement of technologies related to the Olympics, biomedical, and scientific sciences. Appropriate medicine has been designed to implement specific and more specific treatments for specific diseases and patients [42]. The healthcare industry was booming in the pharmaceutical industry. Once again, like the confirmations, text, numbers, photos, and catalogs, any information that lists the large and irregular discovery of various health service management systems lists patient information. At the same time, hospitals were part of several geographical departments in different locations. In different ways, fact provide patient health information from time to time. In response to these problems, Damien is a one-sided solution to healthcare interventions for a marine, vegan-based healthcare management system [43]. The incidence of pediatric and pediatric diseases such as pneumonia and diarrhea are globally challenging. The Patient Demographic and Health Survey (DHS) deportation post from India once again created cesarean section (CBNs) of the day and explored the location factors of childhood diarrhea. Location of freeware tools for DHS data, graphic structure learning with world score-based limitation, and hybrid structure learning algorithms are described. The study identified the outcome of missing values, sample size, and constraints of knowledge based on each of the structure learning algorithms and evaluates their accuracy with multiple scoring functions. [44]. Waring et al. [45] have helped healthcare specialists in the knowledge literature review in the Greater East using automated machine learning (AutoML) with the latest experience of machine learning models “O-Shelf” with limited information data specialization. The possible opportunities and risk of using AutoML in healthcare in the field are also located in the foreground, as well as the demands of AutoML in healthcare in response to the attack. The use of ML techniques has the possibility to improve outcomes of health, reduce costs of healthcare, and demonstrate clinical research. The Greatest Conventions Nowadays, using AI, previously discovered that knowledge can be found in large collections. Clinical oncology data is a start to clinical practice and research with a wealth of multithreaded documents and metadata. Most of our clients include companies and employees. Inadequate interventions, short-term stay, and vision can improve patient care. Incorporating powerful AI algorithms has been instrumental in changing the presentation and common sense of high-intensity radiation oncology. However, this is possible by establishing a clinical scientific community with radiation oncology [46].

### 3.2. Technological Innovations in Healthcare

Blockchain technology, such as the vascularization of inherited traits, router transparency, and identification information, was introduced in 2008 in the Bitcoin cryptocurrency. A wide range of domain-level domains engaged in the health domain. The purpose of this study is to systematically acquire startup publications and evaluate the Turkish position of the use/offer of blockchain to improve processes and services in healthcare, health sciences, and services sanitary [47]. There are some biological processes in which cell regulation and signaling are involved through the assembly of protein complexes. When there is any change occurring through protein-protein interfaces, it will affect the formation of multiprotein complexes. Due to this, sudden change occurs in the cell functions and the development of genetic diseases occurs like cancer and develops drug resistance. These proteins are essential and lead to the formation of many resources for predicting their effects. It should prepare for how mutations affect the structure and body of multiprotein complexes [48]. There are some models under development for the solution of two different problems computationally, to allocate the fund for infectious diseases in the deserts and forests of Africa. Guidance about empirical data collection and theory development for the development in the future is provided [49]. Biomedical research is getting completely changed with big data. The extraordinary advances of automatic data collection of large-scale clinical and molecular data have caused prime challenges to data simplification and analysis, summarized for the evolution of new computational techniques. The development of the system with the efficient use of biomedical big data in particular medicine will need noble scientific and technical creation in which engineering, infrastructure, financial management, and projects will be included. In this study, how the transformation of data-driven techniques provides the probability to address many of these problems has been reviewed, directing the elaboration of the theory on system functions and the generation of technical models and assisting the design of clinical procedures in precision medicine [50].

The article "Influential Usage of Big Data and Artificial Intelligence in Healthcare" was retracted in 2023. Reasons: signs of a paper mill; suspected computer-generated content; unreliable results or conclusions; concerns about the data.

Ear disease and mastoid diseases can be easily handled if early detected with appropriate medical care. However, sometimes, we do not have specialists or we may have comparatively low diagnostic precision if a new way of diagnostic policy is needed, in which deep machine learning can play a noble role. Cha et al. [51] have presented a machine learning model for automatically diagnosing ear disease with the help of datasets having a total of 10544 images which were trained using CNN to categorize internal eardrum and external auditory canal features into 6 categories of ear diseases, which has covered most of the ear diseases.. Inception-V3 and ResNet101 are the learning models which have been chosen for the time training and accuracy, which has an average accuracy of 93.67%. This classifier is trained in various conditions and environments and gives better results of diagnosis, so it is more compatible for the use in a practical environment. For various countries, EQ-5D-3L (three-level EuroQol five-dimensional questionnaire) value sets are entrenched to evaluate the utility of the health state. Before generating these values, analysts gather values for a prechosen health state from a console who represents the public and then use a mathematical algorithm to produce values for 243 states. To estimate the rationality and correctness of both the newer criteria and, earlier, in terms of forecasting of values for all health states and of the values of common health states in specific, preexisting dataset has been used that accommodates VAS (visual analogue scale) values from 126 students while each student has valued all 243 states. A sequence of representations was produced, and eventually, data were designed according to each model. Few of them were used in the past [52]. Related to scientific activity, this study shows a large data depository, containing epidemiology, clinical, and molecular data, which offers research opportunities and is essential to assist scientific activity. The advantages of massive data may contain low-cost collection. Restrictions may contain the cost and difficulty of data storage and processing, which is essential for modern approaches like formatting, analysis, and concerns about security, accuracy, and reliability. It is explained that the source of big data and tools for its analysis can be used to help and diagnose the treatment and management of dermatologic diseases [53]. Diabetes is a condition in which glucose levels are lowered into the bloodstream with a slight delay, causing the inability to metabolize it. When the insulin in the body does not respond properly or if the body does not produce it, this results in diabetes. Serious and long-term health issues are reported. The administration does not really treat electives that include heart pain, lung disorders, skin and liver disorders, nerve damage, and noise damage; quick findings are rare. Thakkar et al. [54] has discussed some valued techniques to excavate in the future and for the diagnosis of diabetes.

Tandon et al. [55] present current issues and opportunities to use blockchain technology to improve health performance. The SLR (systematic literature review) results show that blockchain is being used to create new jobs to improve the standards for the management, distribution, and processing of personal medical records. Implementing the blockchain technology is part of the healthcare system, at verity in the healthcare industry, where the significant value has been added by improving the performance, nearness, advancement of technology, protection, security, and privacy of information management systems. The collection and elaboration of information on public technology has been incorporated by the government and by the real estate companies of the whole world as a strategic solution to alleviate the information of COVID-19 that prevents information. However, the law regarding the end-of-life monitoring system to monitor those who are unable to read the following documents for the help in using the documents of power of the public in the world. EHRs contain valuable information on the progression of Rangatahi's disease and the tragedy of treatment. In the heart failure study, Esther and her colleagues proposed a scheme for extracting short-term sequential samples from CCE data that grading improves phenotype and prediction and is also professional. Brief information on EHR on disease progression and treatment outcomes are given. This article presents a method for representing transient transitional CCE observations up to machine learning. Using clinical data from patients with heart disease, EHR drug transfer and provisional representation from diagnostic and class records for prescribing activities are given [56]. Virtualization (AI) and machine learning are having a real impact in many areas of the healthcare industry. The cancer site is a global phenomenon. Efforts to reduce the chances of accidents should be timely. However, metastatic development, serotonin frequency, and drug inhibition are observed. It is important to find new biomarkers that stimulate group resistance and improve drug delivery to improve carriers to improve carriers [57]. Timeline risk assessment tools for heart failure use a database designed with realistic, one-time clinical document scans and low accuracy. The purpose of this study was to create a comprehensive 30-day plan for unannounced announcements and accurate forecasts for all. All-cause mortality (ACM) connects clinical and clinical information available on the electronic medical record system. There are three predictive indicators for a 30-day unstructured reading or ACM created using a step-by-step method: (a) index admission model, (b) feature-aggregated model, and (c) index discharge model [58]. The study has talked about artificial intelligence that it has the ability to mimic human characteristics, knowledge storage, learning capacity, and so on. There are a majority of techniques which have been already applied in medicine and healthcare, such as the C-statistic model, which was used in North Carolina hospitals as the finest model for the prediction and enhancement of the efficiency of preventive medicine [59].  Table 1 represents some of the existing research work available in the literature.

The article "Influential Usage of Big Data and Artificial Intelligence in Healthcare" was retracted in 2023. Reasons: signs of a paper mill; suspected computer-generated content; unreliable results or conclusions; concerns about the data.

### 3.3. Cardiovascular

Cardiovascular imaging is getting changed with the rise of data science. There are many techniques which have been applied in cardiovascular medicine for exploring different types of diseases, as well as to improve patient care quality and mortality rate. The potential of AI in cardiovascular medicine is tremendous, although ignorance of the challenges may overshadow its potential clinical impact [60]. There are some complexities like efficiency, timing, and missing diagnoses which occur in all stages of the imaging chain. The dependency of AI's applications falls on vigorous data, suitable computational techniques, and tools. While in some areas, it depends on the validation of its clinical application to image sectionalization, automated measurements, and diagnosis. Cardiovascular disease has now accurate imaging combined with big data from the eHealth record and pathology to better characterize the disease and personalized therapy [61]. Research has explored the area and presented studies on the available literature in the area [62, 63].

### 3.4. Big Data and Disease Identification

In daily clinical work, imaging data usage has the ability to improve cancer care by knowing tumor biology and helping in the implementation of precision medicine. For accession of tumor and its microenvironment, radiomics helps in monitoring and evaluating tumor features such as temporal and spatial heterogeneity [64]. Asthma is inconsistent in clinical associations and poor replication of genetic associations. Asthma is not a single disease but a group of similar diseases with some clinical manifestations. Big data for the disease is not providing a solution, just giving information about the disease. Bayesian and frequent approaches make us understand about the ethnology of diseases commonly used in statistical machine learning and can be applied to both big and small data in healthcare research. We need to know about the reality of asthma and not to just give predictions only. We have to get awareness from methodological polemics on data science. The Bayesian and frequent paradigms of the present artificial dichotomies are given. Big data are required to divide the asthma into subtypes to get the solution. Exploiting disaggregated phenotypes and genomic research and the exploration of lung function as an intermediate phenotype. Cohering inductive and deductive statistical approaches to epidemiology pragmatic bayes and unifying graphs are presented [65]. There are techniques and methods by which patients can be classified effectively as those who have asthma and those who do not have those in long-term remission [66]. VA-PODR (Veterinary Affairs Accurate Oncology Data Collection) is a worldwide large repository of well-known data concerned with diagnosed patients of cancer in VA's (Veterans Affairs) department. This data consists of long-term clinical data from the nationwide Veterans Affairs eHealth record, medical photography data, tumor sequencing targets, pathology slides, and the Veterans Affairs central cancer registry as well as CT (computer tomography) scans. A subset of this data storage is available in GDC (genomic data commune) and the TCIA (The Cancer Imaging Archive) [67].

The article "Influential Usage of Big Data and Artificial Intelligence in Healthcare" was retracted in 2023. Reasons: signs of a paper mill; suspected computer-generated content; unreliable results or conclusions; concerns about the data.

The allergic conjunctivitis population has a frequency of 15–20%. However, due to the lack of understanding, the multicause of chronic obstructive pulmonary disease is that the environment, residence, and direct distribution have complex relationships. The benefits of medicine for chronic kidney disease patients and the type of treatment for dementia, as well as the possibilities for other diseases that need to be known by patients that will help patients according to the symptoms and risk factors of the intervention's social empowerment and rehabilitation of people with chronic obstructive pulmonary disease to reduce the body helping to create permanent solutions and prevent the escalation of social ills [68].

In biomedical repositories, the size of somatic genomes is getting increase. So predicting documents related to cancer sets using mathematical algorithms are described. Mining models of conventional gene-based somatic cancer are unhampered by somatic gene ranking and feature extraction due to high computational cost and memory of large datasets. A wide range of characteristics, preferences, and feature squeezing procedures is available, and they are normally deployed in many areas. Each of these procedures tries to extract and squeeze some new irrelevant characteristic features from the trained datasets, having a goal of increasingly accurate results for the newly arranged documented data. Extraction or squeezing of data is an activity of delivering required and related data from a large collection of datasets according to the given information. There are criteria for ranking the information which is sorted as the best results will have the top priority so it will be on the top of the provided list. Experimental results have different cluster sizes with different gene features for clustering of somatic documents. And their generated results prove that the existing model has a high quality of computational clustering [69].

The article "Influential Usage of Big Data and Artificial Intelligence in Healthcare" was retracted in 2023. Reasons: signs of a paper mill; suspected computer-generated content; unreliable results or conclusions; concerns about the data.

## 4. Challenges and Barriers Faced by Healthcare

The healthcare organizations are facing many challenges like analyzing large-scale data. With the rapid increase in healthcare applications, many devices are used to generate verities of data and many of them are used for better analyzing data and for better decision making [70]. The following are the challenges which todays healthcare organizations are facing.

### 4.1. Social Media

Analysts of today's era are giving name to the period that we are living in “an era of fake news” based on the spread of misinformation produced, which may be spread intentionally or unintentionally. As it is affecting all areas and fields of life, it also creates problems and issues in fields related to health, where it may cause to detain or stop effective care, while in some cases, it is menacing the lives of individuals. Wang et al. [71] have exposed the present proof and made it clear in an understandable way; the mechanism of misinformation spreads. The most substantial and considerable topics include misinformation related to vaccination, Zika virus, and Ebola, even though others, such as fluoridation of water, nutrition, cancer, and smoking are also highlighted. Most studies employed content analysis, social network analysis, or experiments, drawing on disparate disciplinary paradigms. Respective systems are used to classify this data based on the result and condition of each sentence [72]. Future research should examine the susceptibility of different sociodemographic groups for misinformation and to understand the role of belief systems on the intention to spread misinformation.

### 4.2. Knowledge about Machines and Technology

Most of the technicians or users of the machines do not have enough knowledge on using the technologies/machines [73]. To overcome this problem, technicians and operators should have sufficient data and knowledge about machines and technology before using it, as most of the machines used in medical and healthcare emit radiation which is quite harmful and dangerous for humans and buildings. The euroCAT infrastructure needs to be implemented as a radiation clinic [8].

### 4.3. High-Power Consuming Technologies

As these artificial machines can perform a complex tasks; many of the technologies operate on large scale in large areas for a long time, which consumes much electric power while there is a big issue of power in most of the developing countries which needs to be solved and adjusted to give plenty of facilities in healthcare.

### 4.4. Expensive

This is the generation of robotics and artificial intelligence which has large significance in the field of healthcare. However, technologies, machines, and data storages, either cloud database or our own database, are mostly not affordable by the organizations because of high prices. By using single-cohort model parameters, we can obtuse the price issues which we are facing and we will face in the future [74]; this will add a significant value to the medical organizations as well as patients in rural areas who cannot afford and do not have access to these technologies.

The article "Influential Usage of Big Data and Artificial Intelligence in Healthcare" was retracted in 2023. Reasons: signs of a paper mill; suspected computer-generated content; unreliable results or conclusions; concerns about the data.

### 4.5. Transformation

A healthcare transformation is a method of sharing thoughts of a company to work on that. It has the importance as the old technology is transforming to a newly developed and evolving technology based on innovation, which may include digital health, eHealth, mHealth, and sensor-based technologies. Such enhancement in health may be significant in identifying diseases on the next level. There are some things which need to be observed before transforming shifting from traditional healthcare to virtual and real-time diagnoses which remains lacking in true evaluation whether these inventions are really improving and overcoming the healthcare quality or not. If any of the new technology is adopted which is not based on evidenced care may risk unintended outcomes like privacy breach, increase in care cost, etc [75]. Distributed ledger technology needs to be implemented to ensure the integrity and authenticity of data produced by embedded systems [76].

The existing literature was studied to know about the details of research available in the area of healthcare based on AI and big data.  Figure 1 represents the details of the literature in the Springer library from various perspectives as given in the figure.

Figure 2 elaborates the details of the search process in the library of ACM.

The library of IEEE was also searched for getting the associated details.  Figure 3 describes the details of the search process for the IEEE library.

Lastly, the ScienceDirect library was tried and the details of the library from various perspectives are shown in Figure 4.

This library was further elaborated and some of the details are shown in Figure 5.

## 5. Conclusion

Big data and AI have revolutionized everything that has brought comfort to people's life in all aspects of daily life. Especially, it is bringing innovative technologies in healthcare systems. It has transformed the conventional and traditional health system to a technological systems in the form of cardiovascular, oncology, ear, asthmatic, allergic, cancer, and or any other diseases. Big data has made it easy to diagnose disease through virtual and real-time systems. The contribution of this paper is to review the present research applicable to mHealth and eHealth where various approaches and models are discussed which use big data for diagnosis and healthcare system. This paper has summarized the current encouraging applications of AI and big data in medical health and electronic health, which have potentially added value to the diagnosis of disease and patient care. The proposed research will help researchers to devise new solutions in the area of healthcare.

The article "Influential Usage of Big Data and Artificial Intelligence in Healthcare" was retracted in 2023. Reasons: signs of a paper mill; suspected computer-generated content; unreliable results or conclusions; concerns about the data.

## Figures and Tables

**Figure 1:** Details of the search process in the Springer library from various perspectives.

**Figure 2:** Details of the search process in the ACM library.

**Figure 3:** Details of the IEEE library from various perspectives.

**Figure 4:** Details of the search process from various perspectives in the ScienceDirect library.

**Figure 5:** Details of the ScienceDirect library.

**Table 1:** Existing research in the area.

S. no.	Title	Year
1	Modeling future price and diffusion in health technology assessments of medical devices	2016
2	Big data effort in radiation oncology	2016
3	Processing and analyzing healthcare big data on cloud computing	2016
4	Decision rules for health system strengthening	2016
5	Use and analysis of big data in dermatology	2017
6	AI in precision cardiovascular medicine	2017
7	Disaggregating asthma	2017
8	Predicting the risk of acute care readmissions among rehabilitation inpatients	2018
9	Selecting health states for EQ-5D-3L valuation studies	2018
10	Modeling asynchronous event sequences with RNNs	2018
11	Map reduce-based hybrid NBC-TFIDF algorithm to mine the public sentiment on diabetes mellitus	2018
12	The trifecta of precision care in heart failure	2018
13	Roadmap for innovation-ACC health policy statement on healthcare transformation in the era of digital health, big data, and precision health	2018
14	Authenticating health activity data using distributed ledger technologies	2018
15	Spread of health-related misinformation on social media	2019
16	Big data analytics for personalized medicine	2019
17	Diagnosis of ear disease	2019
18	AI in cardiovascular imaging	2019
19	Big data visualization in cardiology	2019
20	Big data features, applications, and analytics in cardiology	2019
21	Transitive sequencing medical records for mining predictive and interpretable temporal	2020
22	AI and big data in cancer and precision oncology	2020
23	Electronic health data and machine learning for the prediction of 30-day unplanned readmission or all-cause mortality in heart failure	2020
24	The veteran affair precision oncology data repository	2020
25	Medical big data for P4 medicine on allergic conjunctivitis	2020
26	Somatic cancer gene-based biomedical document feature ranking and clustering	2019
27	Anatomization of data mining and fuzzy logic used in diabetes prognosis	2020
28	Blockchain in healthcare	2020
